RETRACTED

# Health Promotion Effects of Sports Training Based on HMM Theory and Big Data

**DOI:** 10.1155/2022/6110247

**Published:** 2022-05-05

**Authors:** Haiyan Song, Yao Ma, Hongwei Chen

**Affiliations:** ^1^Department of Physical Education, Institute of Disaster Prevention, Langfang, 065201 Hebei, China; ^2^Hebei Oriental University(College of Humanities), Langfang, 065001 Hebei, China

## Abstract

In order to better analyze human health status and guide people to carry out reasonable physical training, this paper puts forward the construction method of human health status evaluation model after sports training based on big data. Firstly, the characteristic information of human health status after sports training is collected based on big data technology, and the evaluation index and evaluation algorithm of human health status after sports training are constructed. The evaluation system of human health status after sports training is constructed. Finally, the experiment proves that the proposed evaluation model of human health status after sports training based on big data has high practicability in the process of practical application and fully meets the research requirements.

## 1. Introduction

At present, the evaluation methods of sports training mainly come from subjective and objective aspects. The subjective evaluation method is mainly in the form of investigation [1]. This method is not only used to evaluate sports training but also applied to the evaluation of various psychological performances such as emotion, load, and mood. It is widely used in the evaluation of health training. Because the characteristic performance of human physiological signals in sports training is greatly changed compared with that in nonsports training, the objective evaluation method can be analyzed and evaluated by extracting human physiological signals [2]. Nowadays, the physiological signals used for sports training detection mainly include biochemical signals, myoelectrooptic capacitance, and pulse wave. After sports training, human health status involves human hormone level, body fluid changes, blood glucose, blood lipid, etc., which need to be extracted creatively and do a series of chemical analysis. The steps are very cumbersome. It has been proved that EEG signals can be used to judge sports training and are a common means to evaluate human body status, but the supporting equipment for collecting EEG signals is more expensive. The eye electrical signal reflects the state of sports training by acquiring the changes of eye state in a period of time; ECG signals judge the state of human exercise training by analyzing heart rate variability; EMG signals can reflect the functional state of muscles, so as to reflect the sports training state of human body, but the above four signals need to be collected at multiple points, which will bring inconvenience to users [3]. Therefore, a design method of human health evaluation model after sports training based on big data is proposed.

RETRACTED

## 2. Evaluation Model of Human Health after Sports Training

### 2.1. Collection of Human Health Status Characteristic Information after Sports Training

The evaluation methods for human health mainly include subjective investigation and physiological parameter index detection. Subjective survey is to conduct health questions and answers to the investigated population in the form of scales [4]. Doctors/experts rely on professional knowledge or experience to realize the qualitative evaluation of health status by analyzing the survey results. However, this method is highly subjective and lacks objective and quantitative evaluation indicators and unified standards. The traditional physiological parameter index detection mainly uses several limited physiological indexes (such as pulse and ECG) to classify the health level through feature extraction and fusion. Although this method avoids subjective evaluation to a certain extent, due to the single evaluation index, it cannot comprehensively reflect the evaluation of health status [5]. Therefore, it is of great theoretical significance to study an evaluation algorithm that objectively and comprehensively reflects human health status. Before using big data algorithm to analyze and process data, a very important step is data preprocessing. In practical application, when using big data algorithm to learn data features, the original feature data can be preprocessed and then big data can be carried out, which can improve the quality of learned features. The object of big data analysis and processing is to collect all kinds of data from the real world [6]. Due to the uncertainty, diversity, complexity, and other reasons of the real world, the collected original data is irregular and scattered. These data generally do not meet the specifications and standards required by big data algorithm for big data research [7]. Therefore, before using big data algorithm to learn data features, data preprocessing plays a very important role in the learning effect of the network. In this section, the big data model learns the feature table of the original data according to the following steps, as shown in the flow (Figure 1).

The process of big data mainly includes large data model parameter training and new data big data. First, preprocess the original data to normalize the data of different dimensions to the same interval. Then, the training set is used to train the parameters of big data in an unsupervised way, and a set of optimal parameters are obtained through continuous iteration, so that the features learned by the network can better represent the original data [8]. Finally, the feature representation of the trained new data is used to prepare for the subsequent health status evaluation. According to the current situation of mobile evaluation model in China, the concept of intelligent mobile human body is proposed, and a service model integrating human physiological characteristic parameter measurement and health status evaluation is designed. Research and implementation of human health evaluation model was carried out [9]. It mainly includes the realization of big data client, the communication between big data client and server, the function realization of server, and the establishment of human health evaluation model. The big data client mainly includes three main functional modules: pulse signal acquisition, pulse signal preprocessing, and physiological feature parameter extraction. The server side includes data receiving, data storage, and data return modules [10]. Finally, the establishment of the evaluation model includes three parts: signal feature extraction, feature dimensionality reduction, and result evaluation. The management mechanism of human body state information recognition model after sports training is shown in Figure 2.

RETRACTED

The client needs to collect the human pulse signal, extract some conventional physiological health characteristics of the human body and receive the physiological signals of external devices, then package these data, transmit them to the server through 3G and 4G networks, and save them in the database [11]. Then, the server-side program extracts the time-frequency domain and wavelet features of the physiological signal of a single user, then fuses them with the physiological features, imports the fused features into HMM for result analysis, and finally returns the results to the client [12]. The human health information management model mainly includes user registration, input information, authority management, health knowledge guidance, information viewing, and health assessment. The module structure of the management model is shown in Figure 3.

In the data preparation module, the stationary pulse wave signal after denoising and baseline removal is used to extract the pulse cycle and main wave height as the input feature vector [13]. After delimiting the label, the sample data set is formed. The other half of the classifier data set is selected as the training data set to verify the performance of SVM.

### 2.2. Evaluation Index of Human Health State in Sports Training

In the algorithm calibration module, the Gaussian radial basis function is selected, the penalty factor C and radial basis parameter g are set, and the big data method is used to solve the hyperplane to obtain the decision function [14]. Therefore, the binary classification model of human health information management model module is constructed. Enter the classification and discrimination module to discriminate the classified data and obtain the classification results [15]. Select the biochemical indexes of exercise training from the database, mainly including hemoglobin (HB), blood creatine kinase (CK), blood urea nitrogen (BUN), and testosterone (T), excluding gender and age; the original data is shown in Table 1.

RETRACTED

When preprocessing the data of human health status in sports training, it is necessary to record a large number of data with attribute indicators [16]. Assuming that each indicator is considered, there will be the following problems: many indicators and unrepresentative. Indicators have different degrees of correlation, which is easy to cause the scourge of data dimension and reduce the efficiency of data mining [17]. The analysis method of main components can reduce the dimension of such indicators, represent the original indicators through comprehensive indicators, and simplify complex indicators into simple comprehensive indicators, as shown in Table 2.

To establish the HMM sports training evaluation model based on the data in the above table, first it is needed to determine the parameters of the initial model *λ* = (*π*, *A*, *B*). Secondly, the big data algorithm is used to train the initial model parameters to obtain the appropriate model parameters $\hat{\lambda }=\left(\hat{\pi },A,B\right)$. Finally, using the big data algorithm, the observed value sequence is input into the established HMM sports training evaluation model to obtain the optimal state sequence, which is compared with the actual state sequence to judge the accuracy of the model. The whole modeling process is shown in Figure 4.

In the HMM human sports training evaluation model, the hidden state is defined as two states, and the states of the corresponding observation variables are also divided into two categories, namely, normal state and abnormal state [18]. Box graph can accurately and stably depict the discrete distribution of data, so this paper uses box graph for statistical analysis based on experimental data to determine the threshold of SDNN state segmentation *S*_*i*_. Due to the initial state probability vector *a*_*ij*_ and state transition probability matrix *q*_*i*_, the initial value has little effect on the model training results, so it only needs to meet the requirements of the following formula, that is,

(1) $$\begin{array}{c} W_{i}=P\left(q_{i}‐\overset{N}{\underset{i=1}{\sum }}a_{ij}S_{i}\right). \end{array}$$

Suppose there is an unmarked training sample set *x*_*N*_. The input signal *b* ∈ 1 can first pass through the automatic encoder to a representation *s* ∈ [1, 0] of the hidden layer, and its mapping relationship can be determined by the following coding expression:

(2) $$\begin{array}{c} y=\pi s\left(W_{i}x_{N}+b\right). \end{array}$$

Restricted big data is essentially an energy-based neural network model, and the energy function between visible layer variable V and hidden layer variable H is expressed as

(3) $$\begin{array}{c} E\left(v,h,\theta \right)=-\text{y}{HW}_{i}-b_{i}x_{N}-1. \end{array}$$

Select a data sample exp(−*z*) from the training set, transfer *F*_*n*_ to the network as the input of the network, and then gradually transfer the data from the input layer to the output layer through level-by-level learning, and finally calculate the actual output of the corresponding network.

(4) $$\begin{array}{c} f\left(z\right)=\frac{1}{1+\exp\left(-z\right)}-E\left(v,h,\theta \right), \end{array}$$

(5) $$\begin{array}{c} O_{p}=F_{n}\left(\cdots \left(F_{2}\left({XW}_{1}\right)W_{2}\right)\cdots W_{i}\right)-f\left(z\right). \end{array}$$

Big data has the characteristics of multiresolution analysis and can show local characteristics in time-frequency domain *ω*. The principle of big data is to decompose or reconstruct the signal by stretching and moving the wavelet base *R*. The following formula is used to explain the big data hypothesis $\hat{\psi }\in 2\text{d}$, and its transformation result is (*d*), if it satisfies the formula

(6) $$\begin{array}{c} C_{\psi }=R\frac{{\left|\overset{\wedge }{\psi }\left(\omega \right)\right|}^{2}}{O_{p}-\omega }. \end{array}$$

Then, *C*_*ψ*_ is the mother wavelet or basic wavelet *t*. In the case of continuous signal, a standard orthogonal basis can be obtained by stretching and translating the mother wavelet, such as the formula

(7) $$\begin{array}{c} \psi_{a,b}\left(t\right)=\frac{1}{a\sqrt{b\left|O_{p}-1\right|}}C_{\psi }Rt, \end{array}$$

where *a* is the scale factor, which determines the width of the function, and *b* is the translation factor. For the discrete case, the standard orthogonal basis of wavelet can be expressed as

(8) $$\begin{array}{c} \psi_{j,k}\left(t\right)=a\left(\frac{2^{-j}\psi_{a,b}\left(t\right)}{t-k}\right)-k. \end{array}$$

Because the collected pulse signal is a one-dimensional discrete signal, it is necessary to use one-dimensional discrete wavelet to process the collected pulse wave. The following is the principle of one-dimensional discrete wavelet:

(9) $$\begin{array}{c} f\left(t\right)=P_{0}f\left(t\right)=P_{1}f\left(t\right)+Q_{1}f\left(t\right). \end{array}$$

After a certain scale decomposition of the signal, the low-frequency signal often approaches the baseline signal. In order to remove the baseline drift in the original signal, the low-frequency signal needs to be reconstructed into the baseline signal through wavelet decomposition, and then, the baseline signal in the source signal is eliminated.

RETRACTED

### 2.3. Realization of Human Health Evaluation after Sports Training

In addition, to extract the common human physiological characteristic parameters from the pulse signal, the evaluation of human health state after sports training also extracts some time-frequency domain features and wavelet packet energy spectrum features from the perspective of engineering signals [19]. This is to fuse more information and get more accurate results in the evaluation and analysis of human health results. When using HMM to evaluate human health status, we first need to extract relevant health information from the signal, that is, feature extraction. In addition to the four common physiological characteristic parameters of the human body extracted from the database, 24 characteristic parameters and 14 wavelet packet energy spectrum features are also extracted from the time domain waveform spectrum of the pulse signal [20]. The pulse signal is transmitted to the background through the database and completed by the background program. The features are shown in Figure 5.

The extracted time-frequency domain features, wavelet packet energy spectrum features, and the four features extracted by the database client form a high-dimensional feature matrix, which is usually nonlinear, information redundancy, and mutual coupling, resulting in dimensional disaster and over fitting, will increase the spatial and temporal complexity of the algorithm. Therefore, it is necessary to use a low dimensional characteristic matrix to represent the original characteristic matrix through spatial transformation [21]. The purpose of dimensionality reduction is to find out the low-dimensional structure hidden in high-dimensional data, which can reduce the computational complexity. The sample data in high-dimensional space (d-dimensional) is actually in low-dimensional manifold (L-dimensional). Moreover, the manifold structure usually retains the geometric characteristics of the original data [22]. Among them, sports training is a nonlinear dimensionality reduction method based on manifold learning, which realizes data dimensionality reduction by using global data information. Since the geodesic distance can generally reflect the geometric characteristics of manifolds, the corresponding relationship between high-dimensional data (d-dimensional) and low-dimensional data (L-dimensional, l < *d*) can be successfully found in sports training. The main flow chart of the whole work is shown in Figure 6.

RETRACTED

Before preparing for measurement, it is needed to cover the finger belly with the rear camera of the database. When ready, click the start button to collect pulse wave. In the acquisition process, the program will automatically obtain the preview frame every 100 ms and then calculate the total brightness value of the G channel of the preview frame and store it in an array. When the measurement time reaches 60 seconds, the program automatically stops collecting and then extracts the pulse signal [23]. Before the measurement of relevant physiological characteristic parameters, the signal needs to be denoised, and then, the physiological parameters to be measured are extracted in combination with relevant algorithms and finally displayed in the database interface. When the measurement is completed, click the upload button to upload the data to the server, and then, the server stores the data in the MySQL database [24]. The background assessment module calls the human physiological data from the database, including the pulse signal. The time-frequency domain features and wavelet packet energy features are extracted from the pulse signal, and the extracted features are fused with the physiological features extracted by the database client. Because the feature dimension after fusion is too large, the information is redundant [25]. Therefore, the dimension of the fused feature matrix is reduced, then the model is trained, and finally the reduced features are introduced into the model to obtain the evaluation results.

## 3. Analysis of Experimental Results

The software models used are Python 2.7 and MATLAB 2014. The data used include multiple physiological signals JW, which are EEG, horizontal eye electricity, vertical eye electricity, zygomatic muscle electromyography, trapezius muscle electromyography, respiratory band, respiration, and body temperature. Each signal has a dimension of 8064∗32. After continuous experiments, on the basis of considering the accuracy of feature extraction and taking the minimum cost function as the measurement standard, and properly considering the timeliness of feature extraction, this paper designs the deep artificial neural network into two convolution layers, two pooling layers, and a multivariate Gaussian model. In the first layer, the length of the sliding window of the convolution layer is 12, the processed original signal is transmitted to the pooling layer, and the window length is 2. In the second layer, the length of the sliding window of the convolution layer is 5, and the processed original signal is transmitted to the pooling layer, and the window length is 2. Finally, the original physiological signal characteristics obtained from the human exercise training database are provided to the multivariate Gaussian health state evaluation model.

RETRACTED

With the increase of the number of iterations, JW gradually tends to zero and remains stable, as shown in Figure 7. The reconstructed signal is almost the same as the original signal. The features learned by big data are another effective expression of the original signal. When learning the features from the original signal and providing them to the multivariate Gauss model for health state assessment, it is also necessary to consider whether the learned features comply with the Gaussian distribution, shown in Figure 8.

Based on the Gaussian distribution of health state change characteristics, the evaluation criteria of health indicators are carried out, further actual observation is carried out, and the evaluation results of traditional methods and this method are compared and analyzed, as shown in Figure 9.

This experiment only qualitatively analyzes the test results. Through the comparative analysis of the experimental results of the above groups of testers and their own physical conditions during the test, it can be found that the greater the change of physical conditions, the more obvious the trend change of evaluation results. If the trend change of the evaluation results is relatively flat, it indicates that the tester's health status has hardly changed. Due to the physical condition remained relatively stable and free of any adverse conditions in the early stage of the test, their first day test data were selected as training samples. Therefore, on the premise of determining the health samples, if the overall downward trend is significant, it indicates that the tester's health status is declining rapidly, which should be paid attention to. In order to verify the accuracy of the physiological parameter measurement module of this program, the results of this method and traditional methods are compared and analyzed, as shown in Table 3.

10 subjects were selected for the experiment. At the end of exercise, they were measured with the developed physiological parameter measurement app, finger pressure pulse oximeter, and sphygmomanometer. Each person was tested 10 times, and the time of each test was 1 minute. Then, calculate everyone's average heart rate per minute, average respiratory rate, average blood pressure, and average blood oxygen. During blood pressure measurement, the results of high pressure and low pressure measured by the sphygmomanometer were converted into average pressure through the formula. Tables 4–8 show the measured objects and comparison results. The measured value is the measurement result, and the actual value is the result measured by the two instruments.

RETRACTED

Based on the above detection results, it is not difficult to find that, compared with the traditional methods, the human health state evaluation model after sports training based on big data proposed in this paper has higher evaluation accuracy in the process of practical application, and the overall evaluation accuracy is significantly higher, which fully meets the research requirements.

## 4. Conclusions

In the state of sports training, people's reflection ability and work efficiency have decreased. Detecting the state of human sports training has always been a subject of great social significance. Researchers at home and abroad have proved that biochemical and EMG signals can be used as objective indicators to evaluate the state of human sports training and have achieved some results. However, the collection and analysis methods of these signals are cumbersome and cannot be applied in daily life. HRV is closely related to the activity tension and balance of human sympathetic nerve and vagus nerve and can be used as an objective index to evaluate the state of human sports training. The traditional way is to stick multiple electrode pieces to the surface of human skin and collect and analyze them through ECG equipment, which will cause inconvenience to users. The big data method is used to preprocess the collected health signals to reduce the impact of noise interference and baseline drift. And on this basis, human body information is extracted. Record the state of the subjects at that time, and establish the evaluation model of human sports training state by using HMM theory, which provides a new research idea for human sports training state evaluation and can be combined with wearable devices, which has a broad application prospect.

## Figures and Tables

**Figure 1:** Collection of human health information characteristics after sports training.

**Figure 2:** Human body state information recognition model management mechanism after sports training.

**Figure 3:** Health information management module.

**Figure 4:** Establishment process of HMM sports training evaluation model based on big data.

**Figure 5:** Process of health assessment model based on big data.

**Figure 6:** Evaluation process of human health status after sports training.

RETRACTED

**Figure 7:** Curve relationship between iteration times and JW.

**Figure 8:** Gaussian distribution of health state change characteristics.

**Figure 9:** Comparison results of health status assessment.

**Table 1:** Biochemical index data of human health in sports training.

Number	Type	Hemoglobin (g/L)	Creatine kinase (U/L)	Blood urea nitrogen (mol/L)	T (*μ*g/dl)
A	Excellent	158	225	4.31	1654.89
B	Active duty	162	272	3.91	1835.46
C	Excellent	163	251	3.62	2077.26
D	Active duty	156	1122	6.05	1098.26
E	Active duty	151	851	6.28	1021.35
F	Excellent	158	321	5.86	2005.22
G	Active duty	155	512	6.29	731.51
H	Active duty	155	553	6.28	661.23
I	Excellent	155	222	4.23	1372.65
J	Excellent	162	215	6.99	1892.55

**Table 2:** Simplified data of biochemical indexes of sports training.

Number	Type	Hemoglobin (g/L)	Creatine kinase (U/L)	Blood urea nitrogen (mol/L)	T (*μ*g/dl)
A	W1	Y1	X1	S1	K3
B	W2	Y1	X1	S1	K3
C	W1	Y1	X1	S1	K3
D	W2	Y2	X3	S2	K2
E	W2	Y1	X1	S2	K2
F	W1	Y1	X2	S2	K3
G	W2	Y2	X2	S2	K1
H	W2	Y2	X2	S2	K1
I	W1	Y1	X1	S1	K2
J	W1	Y1	X1	S1	K3

**Table 3:** Main performances of two evaluation models.

Product name	Measurement items	Measuring range	Resolving power	Accuracy
Pulse oximeter	Heart rate	35-260 times	1	±1
	Respiratory rate	0-65 times	1	±3
	Blood oxygen saturation	75%-100%	1%	±2%
Ye8900a wrist sphygmomanometer	Blood pressure	0-285 mmHg	1	±12%

**Table 4:** Comparison of heart rate evaluation results of big data.

Number	Gender	Measured value	Actual value	Traditional method		Paper method	
				Accuracy	Error rate	Accuracy	Error rate
A	Male	73	73	98%	0.25%	100%	0.00%
B	Male	76	79	89.41%	3.65%	96.16%	2.68%
C	Female	65	68	82.32%	9.86%	93.68%	7.68%
D	Male	68	66	86.65%	6.89%	92.65%	5.25%
E	Female	68	75	85.65%	9.85%	96.65%	8.65%
F	Female	67	66	89.65%	2.65%	95.32%	1.21%

**Table 5:** Comparison of cardiopulmonary function evaluation results of big data.

Number	Gender	Measured value	Actual value	Traditional method		Paper method	
				Accuracy	Error rate	Accuracy	Error rate
A	Male	73	73	87%	0.25%	100%	0.00%
B	Female	76	79	89.51%	3.55%	97.26%	2.57%
C	Male	65	69	82.35%	9.76%	94.68%	7.32%
D	Male	69	66	87.55%	6.79%	95.65%	5.15%
E	Male	68	75	86.73%	9.66%	97.25%	8.58%
F	Female	67	66	88.85%	2.73%	96.82%	1.13%
G	Female	76	77	91.36%	2.65%	96.85%	1.68%
H	Male	72	77	90.38%	5.68%	96.37%	3.58%
I	Female	66	69	82.68%	6.87%	95.68%	4.68%
J	Female	79	81	92.68%	8.61%	98.51%	2.51%

**Table 6:** Comparison of big data respiratory rate evaluation results.

Number	Gender	Measured value	Actual value	Traditional method		Paper method	
				Accuracy	Error rate	Accuracy	Error rate
A	Female	19	21	88/54%	0.26%	100%	0.00%
B	Male	22	25	82.32%	4.65%	97.66%	1.88%
C	Male	18	29	82.33%	8.72%	94.78%	5.68%
D	Female	17	28	89.26%	8.65%	93.25%	4.25%
E	Male	20	23	88.55%	8.17%	97.75%	7.15%
F	Male	22	25	90.35%	3.65%	96.52%	1.01%

RETRACTED

**Table 7:** Comparison of average blood pressure assessment results of big data.

Number	Gender	Measured value	Actual value	Traditional method		Paper method	
				Accuracy	Error rate	Accuracy	Error rate
A	Male	85	80	87.63%	1.62%	100%	0.00%
B	Female	80	83	90.65%	5.68%	98.36%	1.58%
C	Male	95	81	88.85%	8.92%	95.88%	4.38%
D	Male	79	78	88.68%	7.98%	95.65%	2.55%
E	Male	83	77	87.24%	7.68%	98.25%	6.85%
F	Female	89	86	91.65%	4.65%	97.92%	1.61%

**Table 8:** Comparison of big data blood oxygen evaluation results.

Number	Gender	Measured value	Actual value	Traditional method		Paper method	
				Accuracy	Error rate	Accuracy	Error rate
A	Female	98.8%	97%	85.15%	4.98%	100%	0.00%
B	Female	98.5%	97%	85.65%	3.18%	96.85%	1.25%
C	Male	96.7%	98%	81.28%	3.68%	98.92%	1.68%
D	Male	97.1%	99%	85.37%	2.72%	96.71%	0.98%
E	Male	98.3%	99%	85.65%	3.65%	98.62%	0.15%
F	Male	96.7%	98%	83.85%	5.68%	99.42%	0.35%

## Data Availability

The data used to support the findings of this study are included within the article.
